# Explore the Lipid-Lowering and Weight-Reducing Mechanism of Lotus Leaf Based on Network Pharmacology and Molecular Docking

**DOI:** 10.1155/2021/1464027

**Published:** 2021-10-27

**Authors:** Guangjiao Zhou, Xuehua Feng, Ali Tao

**Affiliations:** ^1^Bozhou Vocational and Technical College, Bozhou 236800, China; ^2^College of Pharmacy, Anhui Xinhua University, Hefei 230088, China

## Abstract

**Objective:**

To predict the target of the active ingredient of lotus leaf for lowering fat and losing weight. Explore its multicomponent, multitarget, multipath mechanism.

**Methods:**

Screen the main active ingredients of lotus leaves through the TCMSP database, and use the TCMSP database to predict the potential targets of the active ingredients. Obtain obesity-related targets from the human genome annotation (GeneCards) database. Use Venn software to take the intersection of the two to obtain the effect target of the lotus leaf lipid-lowering and weight-reducing effects. Use Cytoscape 3.6.0 software to construct an effective ingredient-target network. Use the STRING database to construct an intersection target protein interaction (PPI) network, visualize it with Cytoscape 3.6.0 software, and perform network topology analysis to obtain the core target. Use the DAVID database to perform gene ontology (GO) and metabolic pathway (KEGG) enrichment analysis for the above targets. Use AutoDockTools software for molecular docking to verify the binding strength.

**Results:**

A total of 15 main active ingredients such as quercetin, isorhamnetin, sitosterol, and kaempferol were obtained, which can act on 135 targets related to obesity. These targets are significantly enriched in multiple GO and KEGG entries such as hypoxia response, positive regulation of gene expression, response to toxic substances, aging, and positive regulation of RNA polymerase II promoter transcription. Molecular docking shows that flavonoids such as quercetin have better binding to the target protein Akt1.

**Conclusion:**

The lipid-lowering and weight-reducing effects of lotus leaf embody the characteristics of multicomponent, multitarget, and multipathway of traditional Chinese medicine, which provides a certain scientific basis for the screening and in-depth study of the effective ingredients of lotus leaf.

## 1. Introduction

The lotus leaf belongs to the leaf of the Nymphaeaceae plant lotus, which is a medicinal and food homologous plant published by the Ministry of Health [1]. The lotus leaf mainly contains lotus leaf essential oil, lotus leaf alkaloids, lotus leaf polysaccharides, and lotus leaf flavonoids. Lotus leaf flavone is its main active substance, which has the effects of antioxidation, stabilizing blood vessels, dredging blood vessels, and lowering blood pressure. At the same time, it is also a good medicine for weight loss, has the effect of lowering blood lipids, and is often used clinically for the treatment of obesity [2–5]. The fat-lowering and weight-reducing effects of lotus leaves have long been recorded in ancient Chinese medicine books. Due to the complex composition and variety of active ingredients, lotus leaves and their crude extracts have been used for overall functional research for a long time. They all show very good fat-lowering and weight-loss effects [6, 7].

Traditional Chinese medicine has the characteristics of multicomponent, multitarget, and synergistic effects between each component. Network pharmacology is based on the theory of systems biology, and it is a new technology to explain the drug's action and its mechanism [8–10]. Integrating computational virtual computing and network database methods to construct a “medicine-component-target” network, analyze the pathway mechanism and provide guidance for the prediction of the mechanism of traditional Chinese medicine and the multidirectional treatment of diseases [11]. In this study, the network pharmacology method was used to study the characteristics of the multicomponent, multitarget, and multipathway effects of the lotus leaf and to explore the material basis and mechanism of the lotus leaf's lipid-lowering and weight-reducing effects.

## 2. Analysis Method

### 2.1. Screening of Active Ingredients and Targets

Use the Computational Systems Biology Laboratory (TCMSP) to retrieve all the active ingredient data of lotus leaves. It is an important evaluation index for drugs to participate in the process of absorption, distribution, metabolism, and excretion. Taking oral bioavailability (OB) and drug-like properties (DL) as screening conditions, set oral bioavailability (OB) ≥30%, and drug-like properties (DL) ≥0.18 to obtain active compounds that meet the conditions. Obtain the corresponding target points of each active ingredient in TCMSP [12, 13].

### 2.2. Screening Obesity-Related Disease Targets and Lotus Leaf Weight Loss Targets

Search for obesity-related disease targets through the GeneCards database (https://www.genecards.org). Deduplicate, set the correlation score to be greater than 1, and screen out disease targets [14]. Draw a Venn diagram to obtain the intersection of the lipid-lowering and weight-reducing effects of the lotus leaf and the obesity-related targets, which is the pharmacological target of the lotus leaf's lipid-lowering and weight-reducing effects.

### 2.3. Lotus Leaf-Composition-Target-Disease Network Construction

The intersection of the active ingredients of the lotus leaf, obesity, obesity, and the active ingredients obtained from the above screening is taken as the node. Cytoscape 3.6.0 software was used to visually analyze the process of reducing fat and losing weight in lotus leaves. Construct a lotus leaf-component-target-obesity network [15, 16].

### 2.4. Construction of the Protein Interaction (PPI) Network

Enter the lotus leaf lipid-lowering and weight-loss targets in the STRING database (https://string-db.org/). The minimum interaction threshold is set to “highest confidence” (>0.4) to obtain the PPI network and obtain protein interaction information. Use Cytoscape 3.6.0 software to draw the PPI network diagram, and screen out the core targets according to the node degree value [17].

### 2.5. Target Enrichment Analysis and Visualization

Enter the intersection target of obesity and lotus leaf active ingredients in the DAVID database, and perform GO enrichment analysis and KEGG pathway enrichment analysis, respectively. According to the *P* value, the top 10 GO items are selected for analysis. Carry out KEGG enrichment analysis on the signal pathway in which the target participates. According to the *P* value, list the top 10 items for analysis, and draw the core signal pathway diagram [18].

### 2.6. Molecular Docking

Enter the main active ingredients selected under 1.1 into the PubChem (https://pubchem.ncbi.nlm.nih.gov/) database to download the structure of small molecule ligands. Enter the core target protein screened under item 1.2 into the RCSB PDB (http://www.rcsb.org/) database, and download the 3D structure of the target protein. Prepare ligand files and receptor files, and use AutoDockTools software for molecular docking [19].

## 3. Results and Analysis

### 3.1. The Main Active Ingredients of Lotus Leaf

A total of 93 compounds in lotus leaves were retrieved through the TCMSP database, and 15 active ingredients were screened based on oral bioavailability (OB) ≥30% and drug-like activity (DL) ≥0.18. The results are given in Table 1.

### 3.2. Drug-Disease Intersection Target Acquisition

Through the TSMSP database, 189 target proteins of 15 active ingredients in the lotus leaf were retrieved, and the target proteins and gene information were corrected through the STRING database [20]. The GeneCards (https://www.genecards.org) database was searched with “Obesity” as the keyword, and 9,510 obesity-related target genes were obtained. Take 2569 genes with a correlation score greater than 1 and draw a Venn diagram of the targets of the active ingredients in the lotus leaf and the targets of obesity-related diseases. The results are shown in Figure 1. There are 135 intersection targets between component targets and disease targets. The results showed that the lipid-lowering and weight-reducing effects of lotus leaves are related to the 15 active ingredients in lotus leaves and the above 135 targets.

### 3.3. Lotus Leaf-Components-Target-Disease Network Construction

The lotus leaf-components-target-obesity network was constructed by Cytoscape 3.6.0 software. The results are shown in Figure 2.

It can be seen from Figure 2 that the active ingredients and most targets have more interactions. This fully shows that the lotus leaf has the effect of reducing fat and losing weight through multicomponent, multitarget, and multichannel synergistic action. Among the active ingredients, the top 5 active ingredients ranked by the degree value are quercetin, kaempferol, isorhamnetin, O-nornopine, and papaverine. It shows that these ingredients are the main active ingredients of the lotus leaf's lipid-lowering and weight-loss effect [21].

### 3.4. PPI Network Construction and Topology Analysis

Import the obtained 135 intersection targets into the STRING database to obtain the PPI relationship. The results are shown in Figure 3. Figure 3 shows that the network has a total of 135 nodes and 2348 edges. According to the degree value, the top 10 key target proteins are screened out. The results are given in Table 2.

The top 10 targets in terms of the degree value are protein kinase B1 (Akt1), interleukin 6 (IL6), tumor necrosis protein p53 (TP53), caspase 3 (CASP3), JUN protein (JUN), myeloma virus oncogene homolog (MYC), epidermal growth factor receptor (EGFR), epidermal growth factor (EGF), and mitogen activated protein kinase 8 (MAPK8). These targets may be the key targets for the lotus leaf to lower fat and lose weight.

### 3.5. GO Enrichment Analysis Results

A total of 622 GO entries were screened in the DAVID database (*P* < 0.05). GO analysis consists of three parts: biological process (BP), cellular component (CC), and molecular function (MF). Among them, there are 479 BP entries, 44 CC entries, and 99 MF entries [22]. According to the size of the *P* value, the top 10 GO items are listed, respectively, as shown in Figure 4.

It can be seen from Figure 2 that biological process notes mainly include response to hypoxia, positive regulation of gene expression, response to toxic substance, aging, and positive regulation of transcription from RNA polymerase II promoter. The annotation of cell components indicates that the relevant mechanism mainly occurs in the extracellular space, cytosol, plasma membrane, mitochondrion, and extracellular matrix. Molecular functions mainly include enzyme binding, protein binding, identical protein binding, transcription factor binding, and steroid hormone receptor activity.

### 3.6. KEGG Enrichment Analysis

112 KEGG-enriched signal pathways were screened by the DAVID database (*P* < 0.05) [23]. Select the first 10 KEGG signal pathways.  Table 3 provides the details of the pathways.

Analysis shows that the targets are significantly enriched in the hepatitis B signaling pathway, hypoxia-inducible factor-1 (HIF-1) signaling pathway, tumor necrosis factor (TNF) signaling pathway, Chagas disease signaling pathway, and multiple signaling pathways related to cancer. The HIF-1 signaling pathway is shown in Figure 5.

### 3.7. Molecular Docking

Search the three-dimensional structure of the interaction between quercetin (MOL000098), the active ingredient of lotus leaf, and the target Akt1 through the PDB database, download the MOL structural formula of the compound, and import them into the AutoDockTools software, respectively [24]. The binding energy is −6.2. This shows that the receptor and the ligand can bind spontaneously and the result of the binding of quercetin to the target Akt1 target protein (Figure 6).

## 4. Discussion

This study uses the method of network pharmacology to explore the mechanism of the effect of lotus leaf in reducing fat and reducing weight. From the “lotus leaf-components-targets-obesity” network diagram, it can be seen that compounds such as quercetin, kaempferol, isorhamnetin, O-nornopine, and papaverine are important nodes in the network. It is speculated that these compounds may be the material basis of lotus leaf's lipid-lowering and weight-reducing effects. The PPI network of the intersection target of lotus leaf and obesity shows that protein kinase B1 (Akt1), interleukin 6 (IL6), tumor necrosis protein p53 (TP 53), caspase 3 (CASP3), JUN protein (JUN), myeloma virus oncogene homolog (MYC), epidermal growth factor receptor (EGFR), epidermal growth factor (EGF), and mitogen-activated protein kinase 8 (MAPK8) interact with multiple compounds and have high degrees and play a key role in the network diagram. It is suggested that it may be the key target of lotus leaf's lipid-lowering and weight-reducing effects. The GO function is significantly enriched in biological processes such as the positive regulation of gene expression and the positive regulation of RNA polymerase II promoter transcription. KEGG pathway enrichment analysis results show that lotus leaf can play a weight loss effect through the hypoxia-inducible factor-1 (HIF-1) signaling pathway, tumor necrosis factor (TNF) signaling pathway, and multiple signaling pathways related to cancer. The results of molecular docking show that flavonoids such as quercetin have good binding to the target protein Akt1, which provides a strong basis for network pharmacology to predict the reliability of the target. On the basis of network pharmacology, this study discussed the active ingredients of lotus leaf and its multitarget and multipathway characteristics in the process of reducing fat and losing weight. Preliminary explanation of the mechanism of the lotus leaf weight loss effect is provided for the further in vivo and in vitro experimental verification of the lotus leaf weight loss activity and the screening and evaluation of traditional Chinese medicine for weight loss.

## Figures and Tables

**Figure 1:** Venn diagram of the common target of lotus leaf and obesity.

**Figure 2:** “Lotus leaf-components-target-obesity” interaction network.

**Figure 3:** PPI network diagram of the intersection target of lotus leaf and obesity.

**Figure 4:** GO enrichment analysis diagram of the lotus leaf's weight-reducing effect.

**Figure 5:** HIF-1 signal pathway diagram of the lotus leaf weight loss effect.

**Figure 6:** Docking analysis diagram of quercetin and Akt1.

**Table 1:** Basic information of the main active ingredients in lotus leaves.

Number	Id	Compound	OB	DL
1	MOL000098	Quercetin	46.43	0.28
2	MOL000354	Isorhamnetin	49.6	0.31
3	MOL000359	Sitosterol	36.91	0.75
4	MOL000422	Kaempferol	41.88	0.24
5	MOL006405	(1S)-1-(4-Hydroxybenzyl)-2-methyl-3,4-dihydro-1H-isoquinoline-6,7-diol	67.14	0.23
6	MOL003578	Cycloartenol	38.69	0.78
7	MOL007206	Armepavine	69.31	0.29
8	MOL007207	Machiline	79.64	0.24
9	MOL007210	o-Nornuciferine	33.52	0.36
10	MOL007213	Nuciferin	34.43	0.4
11	MOL007214	(+)-Leucocyanidin	37.61	0.27
12	MOL007217	Leucodelphinidin	30.02	0.31
13	MOL007218	Remerin	40.75	0.52
14	MOL000073	Ent-epicatechin	48.96	0.24
15	MOL000096	(−)-Catechin	49.68	0.24

**Table 2:** Key targets of the lotus leaf weight loss PPI network.

Number	Target	Degree
1	Akt1	103
2	IL6	92
3	TP53	89
4	VEGFA	87
5	CASP3	83
6	JUN	78
7	MYC	76
8	EGFR	74
9	EGF	74
10	MAPK8	74

**Table 3:** KEGG channel details.

Number	Pathway	*P* value
hsa05200	Pathways in cancer	2.20*E−*24
hsa05161	Hepatitis B	1.16*E−*20
hsa04668	TNF signaling pathway	1.08*E−*16
hsa05219	Bladder cancer	1.21*E−*16
hsa05212	Pancreatic cancer	6.35*E−*16
hsa05142	Chagas disease (American trypanosomiasis)	1.05*E−*15
hsa04066	HIF-1 signaling pathway	3.19*E−*15
hsa05145	Toxoplasmosis	4.41*E−*14
hsa05215	Prostate cancer	1.54*E−*13
hsa05210	Colorectal cancer	2.55*E−*12

## Data Availability

The data used to support the findings of this study are available from the corresponding author upon request.
